The article "N-Acetylcysteine Improves Inflammatory Response in COPD Patients by Regulating Th17/Treg Balance through Hypoxia Inducible Factor-1α Pathway" was retracted in 2024. Reasons: signs of a paper mill; suspected computer-generated content; unreliable results or conclusions; concerns about the data.

# N-Acetylcysteine Improves Inflammatory Response in COPD Patients by Regulating Th17/Treg Balance through Hypoxia Inducible Factor-1*α* Pathway

**DOI:** 10.1155/2021/6372128

**Published:** 2021-06-29

**Authors:** Xiaopeng Liu, Zhixiong Hu, Haiying Zhou

**Affiliations:** Department of Respiratory Medicine, Jinshan Hospital, Fudan University, Shanghai 201508, China

## Abstract

**Introduction:**

This study was aimed to investigate the effects of N-acetylcysteine (NAC) on chronic obstructive pulmonary disease (COPD) and the change of Th17/Treg cytokine imbalance. *Material and Methods*. A total of 121 patients with stable COPD at the stage of C or D were consecutively enrolled and randomly divided into 2 groups. Patients in the treatment group received NAC granules (0.2 g × 10 bags, 0.4 g each time, 3 times/d) for half a year. The control group was treated with the same amount of placebo therapy. The peripheral blood of the patient was collected and the cytokine, T lymphocyte subsets were detected.

**Results:**

We found the oral administration of NAC could regulate Th17/Treg balance to resist inflammation in COPD patients. Serum testing showed that the proportion of Treg in CD4+ T cells has increased and the Th17/Treg ratio has decreased during the NAC treatment. In vitro studies, we found that NAC regulated Th17/Treg balance through Hypoxia Inducible Factor-1*α* pathway.

**Conclusions:**

Our result could provide new diagnosis and treatment for elderly patients with COPD from the perspective of immunity ideas.

## 1. Introduction

Chronic obstructive pulmonary disease (COPD) belongs to a class of common chronic respiratory diseases characterized by irreversible continuous airflow limitation and high fatality rate, which currently places a huge burden on the world's disease economy [1]. It is associated with both airway and extrapulmonary inflammation, as indicated by increased reactive oxygen species (ROS) levels and proinflammatory markers in peripheral blood. COPD manifests as a series of overlapping phenotypes, including chronic bronchitis, emphysema, small airway disease, and frequent exacerbations. Despite differences in pathology, they share many common but complex pathogenetic processes, including inflammation, excessive oxidative stress, apoptosis, and autoimmunity [2–6].

N-acetylcysteine (NAC) belongs to a class of antioxidants, which has both antioxidant and anti-inflammatory properties. NAC exerts its antioxidant effect by acting directly as a ROS scavenger and a precursor of reduced glutathione [7]. Oral NAC has been shown to affect the body's redox balance through increasing both plasma glutathione levels and lung lavage glutathione levels in patients with stable COPD. However, the clinical effectiveness of NAC in COPD treatment is still controversial. Although it was found in some early studies that NAC had no effect, more recent studies have shown that increasing the dose (1200 mg daily or above) of NAC can reduce the exacerbation of COPD patients and extend the time to the first exacerbation [8–11]. And the most principle of related mechanism is for its antioxidative effect, such as reducing ROS production by alveolar macrophages as well as reducing exhaled H2O2. There are limited data on the anti-inflammatory activity of NAC in COPD patients.

The article "N-Acetylcysteine Improves Inflammatory Response in COPD Patients by Regulating Th17/Treg Balance through Hypoxia Inducible Factor-1α Pathway" was retracted in 2024. Reasons: signs of a paper mill; suspected computer-generated content; unreliable results or conclusions; concerns about the data.

In recent years, lymphocytes, especially CD4+ T cells involved in the pathogenesis of COPD, have become an active topic of research [3, 5, 6, 12]. Studies have revealed that the imbalance between T helper (Th)17 cells and regulatory T (Treg) cells played a vital role in the development and outcome of COPD [5, 12]. Interestingly, though Th17 and Treg cells shared a common requirement for TGF-*β* in their differentiation, they express distinct transcriptional regulators (ROR*γ*t versus Foxp3, respectively) and present opposing functions (inflammatory versus anti-inflammatory). Recent studies have shown that NAC could play as a regulatory role on T lymphocyte subsets differentiation and improve the patient's immune function [13–16]. However, the effect of NAC for T lymphocyte subtype transformation on patients with stable COPD is still unknown.

In this study, we explored the treatment effect of oral NAC on elderly patients with COPD in clinic. And we also determined the change of Th17/Treg balance in peripheral blood of patients who accepted NAC, in order to provide new diagnosis and treatment for elderly patients with COPD from the perspective of immunity ideas.

## 2. Materials and Methods

### 2.1. Ethics Statement

This research was approved by the research ethics committees of Jinshan Hospital Affiliated to Fudan University, China (approval number: Jinshan Medical Ethics Research 2019-13-02). All patients were approached in accordance with the approved ethical guidelines. They had agreed before participating in this study and signed informed consent. All methods used in the study were performed in accordance with the relevant guidelines and regulations developed by the aforementioned ethics committees.

### 2.2. Participants and Trial Design

A total of 121 patients with stable COPD at the stage of C or D based on the Global Initiative for Chronic Obstructive Lung Disease randomly selected from September 2018 to June 2019 were recruited in this research (Jinshan Hospital Affiliated to Fudan University, China). They were randomly divided into two groups. Patients in the treatment group were treated with conventional inhalation of bronchodilators (long-acting anticholinergic drugs (LAMA, tiotropium, 18 *μ*g daily) and oral NAC granules (0.2 g × 10 bags, 0.4 g each time, 3 times/d, Guangdong Baiao Pharmaceutical) for half a year. The control group was treated with conventional airway expansion therapy and the same amount of placebo therapy. No other phlegm-resolving drugs, glucocorticoids, bronchodilators were used during the study. Lung function of each patient was evaluated at the beginning of the study. No significant differences were observed in terms of age, gender, and smoking status of patients between the treatment and control individuals (*P* > 0.05). Clinical data of all individuals are given in detail in Table 1.

The article "N-Acetylcysteine Improves Inflammatory Response in COPD Patients by Regulating Th17/Treg Balance through Hypoxia Inducible Factor-1α Pathway" was retracted in 2024. Reasons: signs of a paper mill; suspected computer-generated content; unreliable results or conclusions; concerns about the data.

### 2.3. Diagnosis of COPD

Diagnosis of COPD was confirmed in accordance with the diagnostic criteria of the Global initiative for chronic Obstructive Lung Disease. The diagnostic criteria for group C were as follows: CAT (COPD assessment test) score <10 or mMRC (modified British Medical Research Council) score was between 0 and 1, the FEV1/pred% is less than 50%, and/or acute exacerbations occur more than 2 times in one year or at least one acute exacerbation occurs which is required in hospital treatment. The diagnostic criteria for group D were as follows: CAT score of 10 or more or mMRC score of 2 or more, FEV1/pred% <50% and/or acute exacerbations ≥2 times per year, or the number of hospitalizations for acute exacerbations is once or more.

### 2.4. Inclusion and Exclusion Criteria for the Study

The inclusion criteria were as follows: (1) patients confirmed as having COPD at stage of C and D; (2) patients who received no antibiotics, glucocorticoids, and theophylline medications within 2 weeks before entering the study; and (3) patients who signed informed consent forms for voluntary participation in the study. The exclusion criteria were as follows: (1) patients with acute exacerbations which may affect the natural process of IL-17 and IL-10 in COPD; (2) patients accompanied by pulmonary interstitial fibrosis, tuberculosis, bronchial pneumonia, and lung cancer; (3) patients with major diseases of nonrespiratory system, such as diabetes, severe cardiovascular and cerebrovascular diseases, and neurological diseases or liver and kidney dysfunction; and (4) patients with mental illness and cognitive impairment.

### 2.5. Blood Samples and Measurements

The peripheral venous blood of the patient was collected in tubes containing ethylene diamine tetraacetate acid (EDTA) in the early morning. The blood samples were immediately centrifuged at 3,000 rpm for 15 minutes after collected, and serum was obtained and stored at −80°C until used. The serum levels of IL-17, IL-10, IL-9, TGF-*β*, TNF-a, and IL-1*β* were determined by using ELISA test kits (R&D Systems, Minneapolis, MN), following the manufacturer's instructions. Briefly, the antibody was diluted to a content of 5 *μ*g/mL, and then, 0.1 mL of that was added into the plate hole and placed at 4°C overnight. The next day, the solution in the plate was discarding, and a 0.1 mL aliquot of the sample was added into the reaction well. Then, place the reaction well into a humid chamber at 37°C for 1 hour. Then, discarding the solution and 0.1 mL of freshly diluted enzyme-labeled antibody was added at 37°C for 1 hour. Then, a 0.1 mL aliquot of substrate solution was added to each well at 37°C for 30 minutes, and 0.05 mL of stop solution was added to each reaction well. The color intensity was measured at a wavelength of 450 nm by using a photometer. The standard curve was plotted based on the concentration of the standard sample and the OD of each well.

The article "N-Acetylcysteine Improves Inflammatory Response in COPD Patients by Regulating Th17/Treg Balance through Hypoxia Inducible Factor-1α Pathway" was retracted in 2024. Reasons: signs of a paper mill; suspected computer-generated content; unreliable results or conclusions; concerns about the data.

### 2.6. Inflammation-Pathway Microarray

Expression microarray analysis was conducted with HWayen inflammation-pathway microarray CSP100. All the procedures and data analysis were performed by HWayan, China.

### 2.7. Flow Cytometry Analysis

Peripheral blood mononuclear cells (PBMCs) were freshly isolated by Ficoll density gradient centrifugation (Pharmacia, Uppsala, Sweden). The isolated PBMCs were washed twice with PBS and resuspended at 106 cells/mL in complete culture medium (RPMI 1640 supplemented with 1% penicillin/streptomycin, 2 mM L-glutamine, and 10% heat-inactivated fetal bovine serum; Gibco BRL, Gaithersburg, MD, USA). For Th17 cells analysis, cells were detected as described previously. For the analysis of Treg cells, a human regulatory T-cell staining kit (BD Pharmingen™, USA) was used to measure CD4+ CD25+ Foxp3+ cells as Treg cells according to the manufacturer's protocol. Briefly, PBMCs were incubated with a cocktail of fluorescein isothiocyanate-conjugated anti-CD4 and APC-conjugated anti-CD25 for 30 minutes at 4°C. After fixation and permeabilization, the cells were blocked by normal rat serum and stained using PE-conjugated anti-Foxp3 for 45 minutes at 4°C. The flow cytometry analyses were performed on a FACS Calibur flow cytometer (BD biosciences, San Jose, CA, USA) equipped with the CellQuest software (BD biosciences). Isotype controls were conducted to ensure antibody specificity.

### 2.8. Western Blot Analysis

The cells were lysed in lysis buffer containing 4% sodium dodecyl sulfate (SDS), 20% glycerol, 100 mM dithiothreitol (DTT), and Tris-HCl, pH 6.8. A total of 30 *μ*g of the supernatant proteins was loaded and separated by 8-15% sodium dodecyl sulfate-polyacrylamide gel electrophoresis. The samples were incubated with primary antibodies overnight at 4°C after the proteins were transferred to a polyvinylidene fluoride (PVDF) membrane (Millipore, 0.2 *μ*m or 0.45 *μ*m, as appropriate), following the electrophoresis [17]. The primary antibodies were used at dilutions of 1 : 1000 for GAPDH (Cell Signaling), 1 : 1000 for HIF1-*α* (Cell Signaling). Then, the membranes were incubated with HRP-conjugated secondary antibodies and visualized with an ECL Chemiluminescent kit (NovexTM).

The article "N-Acetylcysteine Improves Inflammatory Response in COPD Patients by Regulating Th17/Treg Balance through Hypoxia Inducible Factor-1α Pathway" was retracted in 2024. Reasons: signs of a paper mill; suspected computer-generated content; unreliable results or conclusions; concerns about the data.

### 2.9. Statistical Analysis

All analyses were done by using the SPSS software, version 20.0 (IBM Corp., Armonk, NY, USA). Continuous variables were reported as mean ± SD [18]. For two-group comparisons, the independent sample *t*-test was used for normally distributed data [19]. All tests were two-tailed, and a value of *P* < 0.05 was considered statistically significant.

## 3. Results

### 3.1. Oral NAC downregulated the level of IL-17 while upregulated the level of IL-10 in the serum of patients with COPD.

Previous studies demonstrated that increased IL-17 level and decreased IL-10 level in serum were positively correlated with the progression of COPD [20, 21]. To determine whether oral NAC regulated the level of IL-17, IL-10, and other related inflammation cytokine in the serum, we obtained peripheral blood from the patient with COPD for further evaluation. As shown in Figure 1, the level of IL-17 was downregulated in the serum of COPD patients treated with oral NAC, compared to the control counterparts. Conversely, the serum level of IL-10 was upregulated by oral NAC treatment in the COPD patients, compared to the control counterparts (Figure 1). Meanwhile, other proinflammation cytokines, including IL-9, TGF-*β*, TNF-a, and IL-1*β*, were all downregulated. These data demonstrated that oral NAC treatment at a dose of 1200 mg/day was helpful for improving the inflammatory status of COPD patients.

### 3.2. Oral NAC suppressed circulating Th17 cells while promoted Treg cells in the serum of COPD patients.

To further explore the effect of oral NAC, we used IL-17 and Foxp3 as the biomarker of Th17 and Treg cells in the flow cytometry analysis, respectively. As shown in Figures 2(a) and 2(b), the frequencies of Th17 cells were significantly decreased in the peripheral blood of COPD patients in the NAC treatment group than those in the control group (*P* < 0.05). On the contrary, the frequencies of Treg cells were increased accordingly (Figures 2(c) and 2(d)).

### 3.3. Oral NAC rebalances the Th17/Treg ratio.

Constantly, we found that the Th17/Treg ratio was evidently decreased after taking oral NAC in the treatment group from 5.7 to 0.28. This result further proved that NAC could protect patients with COPD by suppressing Th17 immune responses and modulating the Th17/Treg balance in favor of Treg cells. Interestingly, we found that Th17 cells had a negative correlation with Treg cells whether COPD patients took NAC or not (Figure 3).

The article "N-Acetylcysteine Improves Inflammatory Response in COPD Patients by Regulating Th17/Treg Balance through Hypoxia Inducible Factor-1α Pathway" was retracted in 2024. Reasons: signs of a paper mill; suspected computer-generated content; unreliable results or conclusions; concerns about the data.

### 3.4. NAC decreased HIF1-*α* expression of T cells isolated from peripheral blood of COPD patients.

Studies have shown that NAC can downregulate the protein of HIF-*α* by posttranscription mechanism [22, 23]. And specifically, HIF1-*α* is considered as a key regulatory molecule that could directly promote Th17 differentiation by inducing ROR*γ*t transcription and inhibit Treg differentiation through facilitating Foxp3 protein degradation [24]. So, we conducted an inflammation-pathway array to further analyze the pathway related to the change (*n* = 10), and we found that HIF1-a and MAPKp38 exhibited the greatest fold changes in Th17 and Treg cells. Next, we detected the protein and RNA change of HIF1-*α* and p38 expression in Th17 and Treg cells after NAC treatment in COPD patients (*n* = 121). As shown in Figure 4, in the treatment group, western blot revealed that HIF1-*α* significantly decreased in both cells, while p38 had no significant change. The result might reveal that NAC improves inflammatory response in COPD patients by regulating Th17/Treg balance through the HIF1-*α* pathway.

## 4. Discussion

COPD is a type of high-incidence chronic disease in the respiratory system. The occurrence and development of the disease have not been completely studied [1]. In recent years, immune system disorders have been closely related to the cause of the disease. Many researchers have conducted in-depth research in this area. Relevant data showed that, in addition to Th1 and Th2 cells that participated in immune-pathological inflammation, Th17 cells and Treg cells, as subgroups of CD4+ T cells, also played an important role in balancing COPD patients' immune status [5, 20]. Previous researches showed that during the development and acute exacerbation period in patients with COPD, the ratio of Treg and Th17 cells in the peripheral blood has changed significantly, as well as in bronchoalveolar lavage (BAL). The Th17 cells in the serum and Th17/Treg ratio showed a rising trend, but Treg cells were constantly falling. The normal Th17/Treg balance was broken, which led to the appearance of an inflammatory response. At the same time, the increase in Th17 cell level was negatively correlated with the decrease in Treg level, suggesting that the imbalance between these two subgroups might be one of the causes of COPD [21, 25]. Therefore, proper intervention in the Th17/Treg balance of COPD patients was important for the treatment of COPD.

The article "N-Acetylcysteine Improves Inflammatory Response in COPD Patients by Regulating Th17/Treg Balance through Hypoxia Inducible Factor-1α Pathway" was retracted in 2024. Reasons: signs of a paper mill; suspected computer-generated content; unreliable results or conclusions; concerns about the data.

Previous researches have confirmed that NAC had the capability to inhibit the accumulation of neutrophils in the lungs of COPD patients, reducing inflammation, and had a strong expectorant effect [7, 9, 10]. At the same time, NAC had a regulatory effect on immune function and could weaken cytokine activity. Some recent studies had shown that oral NAC could regulate the Th1/Th2 ratio balance, improving the quality of life of COPD patients in groups C and D, increasing lung function to a large extent [26]. Our study showed that the drug could increase the serum interleukin-10 level after oral NAC at a dosage of 1200 mg daily in the treatment group, while the proinflammation cytokine IL-9, TGF-*β*, TNF-a, IL-1*β*, and IL-17 were all downregulated dramatically. Moreover, the proportion of Th17 in CD4+ T cells was decreased, and the proportion of Treg in CD4+ T cells was increased. Therefore, the Th17/Treg ratio was reduced compared with that before diagnosis and treatment. The results suggested that after NAC treatment, the Th17 immune response decreased, the Treg immune response increased, and Th17/Treg tended to back to a new balance, the immune status of COPD patients return to normal. To figure out the mechanism of this effect of NAC, we used inflammation-pathway microarray, western blot, and qRT-PCR to verified that HIF1-*α* might be a key metabolic sensor. In this study, we found HIF-1a was truly significantly downregulated after treatment. Previous studies reported that HIF-1*α* could upregulate IL-17 expression through ROR*γ*t; meanwhile, it also cooperated with ROR*γ*t protein to regulate IL-17A-related genes during Th17 development, thus enhanced the development of Th17 [13, 22]. On the other hand, reports showed that HIF-1 targeted Foxp3 for ubiquitination and proteasomal degradation, using the same ubiquitin ligase system that was responsible for the degradation of HIF-1*α* itself [24]. So, based on the experimental data and result, we proposed a hypothesis that NAC could rebalance the Th17/Treg ratio and improve the immune status of COPD patients through downregulating HIF1-a.

In summary, this study reveals that NAC could affect the Th17/Treg balance in the COPD patients and had a good therapeutic effect for the immune status of COPD patients which might be through regulating the HIF1-*α* expression. By studying the Th17/Treg balance, possible intervention targets may be further found and developed.

## Figures and Tables

**Figure 1:** Oral NAC decreases the level of IL-17 and increases IL-10 in the serum of COPD patients. The level of serum IL-17 in the treatment group increased after oral administration of NAC. The level of serum IL-10 increased in the treatment group after oral administration of NAC. (^∗^*P* < 0.05; ^∗∗^*P* < 0.01; ^∗∗∗^*P* < 0.001).

The article "N-Acetylcysteine Improves Inflammatory Response in COPD Patients by Regulating Th17/Treg Balance through Hypoxia Inducible Factor-1α Pathway" was retracted in 2024. Reasons: signs of a paper mill; suspected computer-generated content; unreliable results or conclusions; concerns about the data.

**Figure 2:** TH17 cell decreased while Treg increased after NAC treatment in the COPD patients. PBMC isolated from peripheral blood and were stained for IL-17 and Foxp3 in order to measure the percentage of Th17 and Treg. (a, b) The percentage of Th17 cells significantly decreased after oral administration of NAC. (c, d) The percentage of Treg cells significantly decreased after oral administration of NAC (^∗∗∗^*P* < 0.01).

**Figure 3:** Oral NAC rebalance Th17/Treg ratio in the COPD patients. (a) The Th17/Treg ratio decreased significantly after oral administration of NAC compared with the control group. (b) Th17 cells had the negative correlation with Treg cells. (^∗^*P* < 0.05; ^∗∗^*P* < 0.01; ^∗∗∗^*P* < 0.001).

**Figure 4:** NAC significantly decreased HIF1-*α* expression of Th17 and Treg cells isolated from peripheral blood of COPD patients. Inflammation-pathway array, western-blot, and qRT-PCR revealed the decreased expression of HIF1-*α* in Th17 and Treg cells in the NAC control group. (^∗^*P* < 0.05; ^∗∗^*P* < 0.01; ^∗∗∗^*P* < 0.001).

**Table 1:** Comparison of baseline data between the two groups.

Term	Control group (*N* = 61)	Treatment group (*N* = 60)	*P* value
Gender (male)	28	30	0.269
Age (mean ± SD)	72.65 ± 7.96	70.89 ± 8.62	0.116
Smoking index	569.07 ± 264.32	592.76 ± 228.54	0.305
mMRC score	2.62 ± 0.85	2.69 ± 0.91	0.277

## Data Availability

All data in this article are available from the corresponding author upon reasonable request.
